# Investigation into Antiepileptic Effect of Ganoderic Acid A and Its Mechanism in Seizure Rats Induced by Pentylenetetrazole

**DOI:** 10.1155/2022/5940372

**Published:** 2022-09-01

**Authors:** Wei Pang, Shuqing Lu, Rong Zheng, Xin Li, Shunbo Yang, Yuxia Feng, Shuqiu Wang, Jin Guo, Shaobo Zhou

**Affiliations:** ^1^College of Basic Medicine, Jiamusi University, Jiamusi, Heilongjiang 154007, China; ^2^College of Rehabilitation Medicine, Jiamusi University, Jiamusi, Heilongjiang 154007, China; ^3^Department of Physical Medicine and Rehabilitation, Qilu Hospital, Cheeloo College of Medicine, Shandong University, Jinan, Shandong 250012, China; ^4^College of Stomatology, Jiamusi University, Jiamusi, Heilongjiang 154007, China; ^5^School of Science, Faculty of Engineering and Science, University of Greenwich, Central Avenue, Chatham ME4 4TB, UK; ^6^School of Life Sciences, Institute of Biomedical and Environmental Science and Technology, University of Bedfordshire, Luton LU1 3JU, UK

## Abstract

Ganoderic acid A (GAA) exhibited neuron protection in *in vitro* epilepsy study, but no study has been done *in vivo*. Rats were administered (i.p.) pentylenetetrazole daily for 28 days to induce seizure. Rats with grade II or above of epileptic score were divided into three groups and given placebo, sodium valproate, or GAA treatment, respectively, for 7 days. The electrical signals of brain were monitored with electroencephalography (EGG); epileptic behavior was assessed using the Racine scale; morphological changes and apoptosis rate of cortical neurons were assessed with H&E staining and TUNEL staining, respectively. Protein expression of calcium-sensing receptor, p-ERK, p-JNK, and p-p38 in hippocampal tissue and Bcl-2, cleaved caspase-3, and Bax in cortical tissues was observed by Western blot and immunohistochemistry assay, respectively. After GAA treatment, apparent seizure-like EEG with significant arrhythmic disorder and spike waves was reduced or disappeared, and wave amplitude of EEG was reduced significantly. GAA showed similar effect with sodium valproate treatments on epilepsy. There were an apparent improvement of the epileptic behavior and a significant increase in the epileptic latency and shortening of the epileptic duration in the treatment group compared to control. GAA treatment ameliorated the nuclear pyknosis of neurons which appeared seriously in the epilepsy group. GAA treatment significantly reduced the cortical neuron apoptosis of epilepsy and the expression of calcium-sensing receptor, p-P38, p-JNK, cleaved caspase-3, and Bax but increased the expression of both p-ERK and Bcl-2. In conclusion, GAA treatment showed strong antiepileptic effect by decreasing apoptosis in cortical neuron and the expression of calcium-sensing receptor and stimulating the MAPK pathway.

## 1. Introduction

There are approximately 70 million people suffering from epilepsy in the world which can be caused by the abnormal discharge of brain neurons due to brain injuries, such as trauma, stroke, intracranial infection, and medical, personal, genetic, and social factors [1, 2]. Up to 90% of patients with epilepsy are living in low income and poor medical conditions [3]. Epilepsy generally cannot be cured and sometimes cannot be controlled by common drugs, e.g., sodium valproate; thus, it seriously affects patients' health and quality of life [4]. Therefore, finding new therapeutic agents is urgently needed.

*Ganoderma lucidum*, a kind of fungus, belongs to the Basidiomycete, Polyporaceae. *Ganoderma lucidum* is widely used to promote health, and it contains compounds such as triterpenoids (ganoderic acids), polysaccharides, sterols, and alkaloids with pharmacological activities. These components can regulate the nervous system and immune system, improve hypoxia tolerance and scavenge free radical, and protect liver function [5]. We have demonstrated the antiepileptic effects of *G. lucidum* in *in vitro* and *in vivo* studies [6–8]. We also found that ganoderic acid A (GAA) reduced the apoptosis in primary hippocampal neurons cultured in medium without magnesium, an *in vitro* epileptic model, but no study on neuroprotection has been done *in vivo* [9]. Thus, this study tested the antiepileptic effect of GAA in an epileptic rat model.

GAA is one of the 140 triterpenoids isolated from *G. lucidum* [10, 11]. GAA has been shown to inhibit cancers of the liver, lung, and kidney, improve insulin resistance, and exhibit anti-HIV activities [12–18]. For instance, after 5 weeks of treatment with GAA (10 mg/kg), the volume of anaplastic meningioma was significantly reduced, and the overall survival rate of mice was improved [12]. GAA can significantly inhibit the invasion and migration of U251 glioblastoma multiforme cells with dose- and time-dependent effects [19]. GAA significantly inhibits the PI3K/AKT pathway by reducing the phosphorylation of AKT, mTOR, and cyclin [19].

The activation of calcium-sensing receptor (CaSR) has been linked to neuron damage in epilepsy and has attracted research interest recently [20–22]. CaSR is distributed in the digestive system, cardiovascular system, etc. and exhibits the ability to regulate gastrointestinal motility, bone metabolism, and kidney function. It is also found in the central nervous system but with limited information on its role in epilepsy [23–30]. CaSR participates in the maintenance of Ca^2+^ homeostasis, as well as the regulation of brain growth and development, cell proliferation, and differentiation, maintenance of membrane potential, and ion channel switching [31–33]. CaSR has also been highly expressed in the hippocampus of epileptic rats [26], and its genetic mutation is related to idiopathic epileptic syndrome [34–37]. Also, there is a positive link between CaSR and the mitogen-activated protein kinase (MAPK) pathway; for example, the overexpression of CaSR can cause epilepsy by affecting the expression of proteins linked to the MAPK pathway.

The effect of GAA on epilepsy and the underlying molecular mechanism *in vivo* have not yet been reported. Therefore, in this pilot study, the effect of GAA on electroencephalography (EEG), epileptic behavior, histological changes, and apoptosis of brain tissues was investigated in an epileptic rat model induced by pentylenetetrazole. The workflow of the study is listed in Figure 1. The aim is to test antiepileptic effect of GAA and provide a theoretical target of GAA on the calcium-sensing receptor and MAPK pathway in order to pave the way for its use in epilepsy treatment.

## 2. Methods

### 2.1. Chemicals

Sodium valproate and pentylenetetrazol (PTZ) were bought from Sigma-Aldrich (MO, USA). GAA (purity was ≥95%) was bought from Dalian Meilun Biotechnology Co., Ltd. (Dalian, China). Antibodies against CaSR, Bcl-2, and Bax were obtained from Proteintech Group, Inc. (Wuhan, China). Caspase-3, p-JNK, p-ERK, and p-P38 were purchased from Cell Signaling Technology, Inc. (Danvers, MA, USA). The TUNEL apoptosis kit was bought from Boster Biological Technology Co., Ltd. (Wuhan, China).

### 2.2. Animal Experimental Design

The Research Ethics Committee of Jiamusi University approved this study (no. jmsukf-2020006). Animals were cared and handled by a specially trained technician on rats in accordance with the guideline of laboratory animal's study by the Chinese Ministry of Science and Technology. A total of 48 healthy male Sprague-Dawley (SD) rats, weighing 180 ± 20 g, were bought from the Liaoning Changsheng Biotechnology Co., Ltd. (Benxi, China), and three rats were raised in each cage away from strong light and noise in the lab of Animal Center of Jiamusi University. The lab has a controlled temperature of 21 ± 2°C, relative humidity of 30–70%, and day-night period of 12/12 h. They had free access to food and water. After one-week adaptation, rats were randomly divided into four groups: control group, epilepsy group, valproate group, and GAA group, with 12 rats in each group. The rats in the epilepsy group, sodium valproate group, and GAA group were administered PTZ injection intraperitoneally (i.p.), with a subconvulsive dose of 35 mg/kg (100 mg of PTZ dissolved in 10 mL saline) at 8-10 am once a day for 28 days according to previous [26] and our studies [38]. The rats in the control group were given the same volume of saline (i.p.). EEG was assessed (see Section 2.3); together with the EEG changes, rats also appeared as grade II for more than 5 consecutive days during this period and were used for the study. From day 29 to day 35, the rats in the control group, epilepsy group, sodium valproate group, and GAA group were given placebo (saline+5% DMSO), sodium valproate (200 mg/kg, dissolved in saline), and GAA (10 mg/kg, dissolved in 5% of DMSO with a concentration of 30 mg/mL) by intragastric administration at 8-10 am once a day, respectively [39]. On day 36, except the control group, the other three groups were administered PTZ (35 mg/kg) again to induce the kindling epilepsy, and their behavior was observed. Then, rats were euthanized with pentobarbital sodium (i.p. 300 mg/kg body weight, dissolving to concentration of 3% in phosphate-buffered saline). Until the signs of ataxia (stumbling, falling, and crossing feet) appeared following injection, the rats were given transcardiac perfusion and the cerebral hemispheres were removed. Half of them (6) were fixed in 4% paraformaldehyde solution, and the others were stored in liquid nitrogen.

### 2.3. Electroencephalography (EEG) Assessment

Rats were given with isoflurane with 5% for induction and 1%–2% for maintenance their general anesthesia. Then, three stainless-steel screw electrodes, with a diameter of 1.2 mm, were individually implanted into the rat's bilateral temporal lobe and the right frontal lobe which are used as a reference electrode. EEG was recorded for up to 90 min using Mfile software. All successful modeling rats were monitored at baseline and after treatment.

### 2.4. Criteria for Epileptic Seizure Grading

Detailed grading of convulsion was based on the Racine scale [40]. It was scaled as in the following: 0: no response; 1: immobilization; 2: partial myoclonus, e.g., nodding head; 3: whole body myoclonus; 4: rearing tonic seizure and multilimb twitches; and 5: generalized persistent tonic-clonic seizures, wild rushing, and jumping [41]. Only rat with five consecutive seizure scores of grade II or above was considered a successful chronic epileptic model [40]. The seizure latency (time difference from the completion of the last seizure to the start of the next one) and seizure duration (from reaching the Racine score of grade 1 to end of the seizure) were analysed.

### 2.5. Hematoxylin-Eosin (H&E) Staining

The rat brain tissues fixed with 4% paraformaldehyde were cut into 4 *μ*m sections and stained with H&E as described previously [42], and the histological structure was observed using a 400x microscope (Nikon ECLIPSE Ni, Japan). Damaged neurons from 6 observed optical fields per rat were counted and used for the statistical analysis among groups.

### 2.6. TdT-mediated dUTP Nick-End Labeling (TUNEL) Assay

The TUNEL apoptosis assay was based on its commercial company manual and our previous study [38]. The results were observed with a fluorescence microscope (OLYMPUS BX51, Japan), and images of a bright-field microscope were taken. The apoptosis rate was calculated by using the number of positive cells to total cells in the same area (%).

### 2.7. Immunohistochemistry (IHC) Staining

The method was based on our previous study with some modification [5]. Paraffin sections of rat cortical tissue were routinely dewaxed and hydrated. The endogenous peroxidase inhibitor was added and incubated for 10 min and then rinsed with distilled water. The sections were put into citrate antigen retrieval solution and heated for 2 min in a microwave oven. Then, blocking buffer with 5% BSA was used. Drops of primary antibody (Bax, 1 : 100; caspase-3, 1 : 1000; or Bcl-2, 1 : 300) were added and stored at 4°C overnight. The following day, the sections were incubated at 37°C for 30 min first and then washed with PBS. The biotin-labeled goat anti-rabbit IgG (second antibody) was added and incubated for 30 min at 37°C. After washing, drops of DAB chromogen were dripped on the sections (the degree of staining was monitored with regular microscopy). Sections were then stained with hematoxylin.

### 2.8. Western Blot Analysis

The Western blot method was based on our previous study with some modification [5]. It was used to test the expression of CaSR, p-ERK, p-JNK, p-p38, Bcl-2, Bax, and caspase-3 in rat brain cerebral cortex or hippocampal tissue. Briefly, the tissue was homogenized, and the supernatant was collected (12,000 rpm, 10 min, at 4°C). The protein concentration was measured by a BCA assay. A 10 mg of protein sample was loaded and separated by SDS gel electrophoresis. The proteins separated from the gel were transferred onto PVDF membranes which were then blocked at 37°C in a TBS solution for 1.5 h. The concentrations of the primary antibody used for the incubation were 1 : 1000 for CaSR, p-ERK, p-JNK, p-p38, Bcl-2, Bax, and caspase-3 and 1 : 5000 for GAPDH. After they were incubated overnight at 4°C, the membrane was washed 3 times with a solution with TBST. Then, alkaline phosphatase-conjugated IgG (secondary antibody) was added and then washed 3 times with a TBST solution. When the protein bands appeared, then the images were taken. GAPDH was used as an endogenous protein for normalization.

### 2.9. Statistical Analysis

SPSS software (version 23; IBM Corp., Armonk, NY, USA) was used for statistical analysis. Values are expressed as the mean ± SE. Student's *t*-test or one-way ANOVA followed by a post hoc analysis (Tukey test) was used for group comparisons. Significant statistical differences were considered when *p* < 0.05 and *p* < 0.01.

## 3. Results

### 3.1. Effect of GAA on the EEG

There were no significant waves and pattern difference in the control group at baseline and treatment. However, significant arrhythmic disorder and spike waves were observed in the epilepsy group (Figure 2), and the appearance of burst suppression episodes was observed in the GAA group. For EEG of baseline, seizure-like EEG in PTZ-induced seizure model was observed in the B, C, and D group. After treatment, significant arrhythmic disorder and spike waves were still observed in the B group, but they were dramatically reduced in C and D groups (Figure 2), and their wave amplitude of EEG in the GAA treatment group was reduced significantly compared to that in the epilepsy group (Figure 3).

### 3.2. Effect of GAA on the Rat's Epileptic Scores

After rats were given PTZ injection intraperitoneally, they started frequent blinking, staring, rhythmic nodding, tail flick, and clonic convulsion of forelimbs within 10-30 min of the injection. After 30 min, the forelimbs of rats were rigid and left the ground. In grade V epileptic seizure, the rats showed limb and body rigidity, jumping, and falling. Rats with 5 consecutive times of grade II or above seizures met the standard of epileptic kindling. There was no seizure in the control group. The successful epileptic kindling model was also confirmed by the EEG monitoring (see Figure 2). During the 7-day treatment with GAA or sodium valproate, the epileptic behavior at day 35, in both the GAA and sodium valproate groups, was much reduced on the rat's epileptic scores, but there were no statistically differences compared to the epileptic model group. However, the seizure latency of the rats in both sodium valproate and GAA groups was significantly increased, but the duration of seizure symptoms was significantly lower than that in the epilepsy group (*p* < 0.05) (Figure 4).

### 3.3. Effect of GAA on Histopathological Changes

Figure 5 shows the morphology of cortical tissues. In the control group, the neurons of the cerebral cortex were normal in shape with good order and good structure with the full cytoplasm. In the epilepsy group, nucleus pyknosis or lysis occurred, the cell structure was destroyed, and the shape was changed. Compared with the epilepsy group, the degree of damage of cells in both the GAA group and sodium valproate group was less severe, and the cell structure was well improved. Results show that the GAA treatments significantly reduced the damaged neurons compared with the epilepsy group without given treatment (Figure 5(e)).

Morphology of hippocampal tissues is shown in Figure 6. The neurons of the hippocampus in the control group were arranged in good order without abnormal morphological changes observed. However, in the epilepsy group, a large number of neurons in necrosis and dissolution appeared, neurons were not arranged in good order, and severely damaged cells were observed. In both the GAA group and sodium valproate group, hippocampal neurons are arranged more orderly than those in the epilepsy group. There is a significant increase in damage neurons in the epilepsy group compared to the normal group, but both the GAA group and sodium valproate group did not statistically reduce the damaged neuron rate, even though there is an apparent reduction.

### 3.4. Effect of GAA on the Apoptosis and the Proteins' Expressions Related to the Mitochondrial Apoptosis Pathway

The apoptosis in rat cerebral cortex tissue stained by the TUNEL technique is shown in Figure 7, where the brown-stained nuclei are apoptotic cells. The apoptosis rate was calculated as the total apoptotic neurons to total neurons in six observed fields. The apoptosis rate in the epilepsy group was significantly highest compared to that in other groups, while treatment with both sodium valproate and GAA significantly reduced the apoptosis rate significantly (*p* < 0.01). The expression of Bcl-2 in the IHC assay is presented in the IHC micrograph (Figures 8(a)–8(d)), and its level of the Western blot assay was decreased significantly in the epilepsy group compared with the control group (*p* < 0.01, Figure 8). However, compared with the epilepsy group, the expression level of Bcl-2 protein was significantly increased in both sodium valproate and GAA groups (*p* < 0.05, respectively).

The expression of Bax protein of cortical tissue is shown in the IHC micrograph (Figures 9(a)–9(d)), and its expression level in hippocampus tissue was increased significantly in the epilepsy group compared with the control group (*p* < 0.05, Figure 9(e)) in the Western blot assay. Compared with the epilepsy group, the expression level of Bax protein in the Western blot assay was significantly decreased in both the GAA group and sodium valproate group (*p* < 0.05, respectively). The expression level of caspase-3 appeared at 17 kDa which is cleaved caspase-3, and it was significantly elevated in the epilepsy group compared with the control group but decreased significantly after both sodium valproate and GAA treatments (*p* < 0.05, respectively, Figure 10).

The expression level of CaSR in hippocampus tissue was increased in the epilepsy group compared to the control group (*p* < 0.05), but its expression was decreased in both the sodium valproate group and GAA group compared with the epilepsy group (*p* < 0.05, Figure 11(a)). The expression level of p-ERK in hippocampus tissue was decreased in the epilepsy group compared to the control group (*p* < 0.01, Figure 11(b)), and its expression was increased in both the sodium valproate group and GAA group compared with the epilepsy group (*p* < 0.01). The expression level of both p-JNK and p-P38 in hippocampus tissue was elevated in the epilepsy group compared to the control group (*p* < 0.05 and *p* < 0.01, respectively); however, their expressions were decreased in both the sodium valproate group and GAA group compared with the epilepsy group (*p* < 0.05 and *p* < 0.01, respectively, Figures 11(c) and 8(d)).

## 4. Discussion

This study established an epilepsy rat model by administration of PTZ daily for continuous 28 days, and those with successfully induced grade II or above of Racine scale were selected and EEG monitored. Then, they were given GAA treatment or placebo treatment for 7 days, and the antiepileptic effect of GAA was monitored by behavior improvement and histological changes. Finally, the molecular biomarkers were assessed by the expression of CaSR, as well as the proteins in the MAPK pathway, e.g., p-JNK, p-P38, p-ERK, Bcl-2, Bax, and cleaved caspase-3 in brain tissue.

PTZ, a GABA-A receptor antagonist, can induce generalized seizure. It can be a mild seizure without convulsion, a tonic-clonic seizure, or an acute severe seizure based on the dosage and frequency given. This model has been widely used in epilepsy research, for screening antiepileptic drugs or anticonvulsant candidates and investigation of neuronal damage after seizure, as the histological changes observed in this model are similar to the brain changes of patients with epilepsy [41]. The epilepsy model was successfully established by administration of PTZ daily for 28 days. Seven-day treatment with GAA and extra PTZ challenge at day 36 both showed the dramatic amelioration of epileptic behavior by GAA treatment to a similar extent as sodium valproate treatment, even though neither showed statistically significant differences compared to the epileptic control group. This indicates that the treatment time should be increased further. However, the latency was increased dramatically, and duration of seizure was decreased significantly; both showed the efficacy of the GAA treatment.

The hippocampus is the key damaged area for chronic epilepsy. The most common damage is the hippocampal angle sclerosis which can originate from vascular disease or hypoxia, loss of nerve cells at the lesion, and proliferation of glial cells and fibers. Another damage area is the cortex where abnormal cells and gliosis appeared at the edge of the cerebral cortex. The degree of cell damage varies. In severe cases, dead cells are replaced by scar tissue and gliosis. In mild cases, only local blood supply disorders or tissue structure disorders are present. Our results showed that neurons in the cortex and hippocampus of the epilepsy group were most seriously damaged by PTZ treatment. In the epilepsy group, the damage was more serious, but GAA and sodium valproate could alleviate the damage by pathological assessment. GAA treatment clearly reduced nucleus pyknosis and lysis occurring in the epilepsy group and restored the neuron histology structure both in cortex and hippocampal tissues. The intervention effect of GAA was comparable to that of the first-line antiepileptic drug, sodium valproate.

Moreover, TUNEL results showed that the apoptosis of neurons in the epilepsy group was the most serious in the cerebral cortex of rats. However, after GAA treatment, the neuron apoptosis rate was reduced significantly, even more than that of the sodium valproate group. The detection of cleaved caspase-3 indicates cell death induction, while its decrease indicates reduction in apoptosis in both cancer and Alzheimer's disease [43]. In this study, GAA treatment decreased the level of cleaved caspase-3 which is consistent with TUNEL results and our previous results of an *in vitro* study [9]. GAA has also shown protective effects via its antiapoptotic role in kidney cyst, intestinal epithelial injury, colitis, and other diseases by inhibiting the MAPK pathway or promoting the apoptosis of cancer cells by enhancing the expression of the MAPK pathway [44, 45].

The expression of CaSR in brain tissue of epileptic rats was increased, accompanied by cell injury and apoptosis [21, 22]. The overexpression of CaSR induces the activation of JNK and p38 in the MAPK signal transduction pathway and promotes cell apoptosis in myocardial and brain tissues; meanwhile, the activation of the p-ERK in the ERK pathway has exhibited protective effect on myocardial and brain tissue cells [20, 22, 26, 46]. Our results showed that protein expression of p-JNK and p-p38 in the hippocampus tissue of epileptic rats increased significantly, and there was a significant increase in CaSR expression in the epilepsy group compared with the control group, while the expression of p-ERK was decreased. GAA treatments reduced the expression of CaSR in the hippocampus, downregulated the expression of p-JNK and p-p38 in the MAPK pathway, and upregulated the expression of p-ERK. There was no significant difference between the GAA group and sodium valproate group. These results indicate that GAA can change the expression of related proteins in the MAPK signal transduction pathway, inhibit nerve cell apoptosis, and protect brain tissue by decreasing the expression of CaSR protein in brain tissue of epileptic rats. Moreover, GAA showed significant effect comparable with sodium valproate, the first-line antiepileptic drug.

Calcium overload can speed up the apoptosis and cause mitochondrial damage [47–49]. Previously, we found calcium overload in cultured epileptic neurons, while *G. lucidum* polysaccharides can inhibit the intracellular calcium accumulation by stimulating the expression of CaMKII to inhibit epileptic effect [50]. The activation of CaSR leads to intracellular calcium overload and causes mitochondrial damage via changing the mitochondrial membrane permeability and disintegration [47]. It has been confirmed that the expression of CaSR is increased in the apoptosis process of the cardiomyocytes of epileptic rats [20].

The expression levels of Bax, cleaved caspase-3, and CaSR are higher in spontaneously epileptic rats while the trend of Bcl-2 expression was opposite with Bax and cleaved caspase-3 [51]. Activation of CaSR can upregulate the expression of the proapoptotic protein Bax but downregulate the expression of the antiapoptotic protein Bcl-2 on the mitochondrial outer membrane, then promote the mitochondrial disruption and cytochrome C release, and further activate caspase-9 and caspase-3 [52, 53]. This is involved in the activation of the JNK/p38 factor in the MAPK signaling pathway, regulating MAPK cascade reaction, thus causing cell damage and apoptosis [54–56]. Both Western blot analysis and IHC analysis found that in the brain tissue of rats, the expression of Bax and cleaved caspase-3 in the epilepsy group was higher than that in the control group, and the expression of Bcl-2 protein which inhibited apoptosis was decreased, which was consistent with the study of Wang [20]. In the GAA group and valproate group, the expression of Bax and cleaved caspase-3 was decreased, and the expression of Bcl-2 protein was increased. This suggests that GAA could decrease the protein content of both proapoptotic proteins Bax and cleaved caspase-3 and increase the content of the antiapoptotic protein Bcl-2 by decreasing the expression of CaSR. While the pathophysiological mechanism of cell damage and apoptosis induced by epilepsy has not been fully elucidated, this and other studies have shown that the activation of CaSR is indeed involved in epilepsy-induced cell damage and apoptosis. Both Kapoor et al. and Delgado-Escueta et al. have shown that genetic error mutations in CaSR are associated with idiopathic epilepsy syndrome [34, 35]. Gene mutation of CaSR can change the abundance of receptors in the plasma membrane, strengthen the activation of related signaling pathways, and alter the regulation of the central nervous system to induce epilepsy [36, 37].

The antiepileptic effect of GAA may be related to the intervention time and dosage [57]. In the treatment of epilepsy, patients often need long-term antiepileptic drug treatment with adjusted dosage based on the degree and frequency of seizures. In this study, a medium dose of GAA intragastric intervention for 7 days due to the cost of GAA exhibited antiepileptic effect similar to sodium valproate, even though there was no statistically significant reduction in the epileptic scores in either treatment group. A follow-up study can prolong the treatment time of GAA to observe the effect of administration time on its antiepileptic effect.

This study did not examine the toxicity and side effects of GAA and sodium valproate, but it was reported that sodium valproate had hepatotoxicity with higher vacuolar degeneration on PZT-induced chronic epileptic rats. However, 10 mg/kg GAA did not cause any hepatotoxicity in mice with meningioma for 5 weeks [12]. In addition, this study did not detect the blood concentration of GAA in epileptic rats and could not adjust the dosage according to the blood concentration of GAA; the study did not compare the different intervention doses of GAA. Future studies of the antiepileptic effect of GAA will focus on the above problems in order to determine the optimal intervention dose and further clarify the antiepileptic effect and mechanism of GAA.

## 5. Conclusions

In conclusion, this pilot study explored the antiepileptic effect of GAA and its molecular mechanism. GAA showed antiepileptic effect by ameliorating epileptic behavior and brain tissue damage by epilepsy. The neuroprotective effects may be via decreasing apoptosis and CaSR expression as well as through the MAPK pathway by decreasing the expression of p-JNK, p-p38, Bax, and cleaved caspase-3 and increasing the expression of p-ERK and Bcl-2. This pilot study paved the way for the further study of its use in antiepileptic treatment.

## Figures and Tables

**Figure 1:** Workflow of the study. Rats were divided into 4 groups; three of them were administered (i.p.) to induce seizure; then, they were given treatment with placebo (normal group), placebo (epilepsy group), sodium valproate (epilepsy treated group), or GAA (epilepsy treated group), respectively. Electroencephalography (EGG); epileptic behavior was assessed, and morphological changes and apoptosis were tested. Protein expression of calcium-sensing receptor, p-ERK, p-JNK, p-p38, Bcl-2, cleaved caspase-3, and Bax in brain tissues was observed by Western blot and immunohistochemistry (IHC) assay, respectively.

**Figure 2:** Representative EEG of a group of rats at baseline (a) and treatment (b). A–D represent groups of control, epileptic model, sodium valproate, and GAA, respectively.

**Figure 3:** The wave amplitude of EEG in each group before and after treatment. ^∗∗^*p* < 0.01 vs. control group, ^##^*p* < 0.01 vs. epilepsy group, and ^#^*p* < 0.05 vs. epilepsy group.

**Figure 4:** The latency of seizure (min) and the duration of seizure (min) of rats from three groups. They are epilepsy, sodium valproate, and GAA treatment groups. The seizure latency is the time difference from the completion of the last seizure to the start of the next one; seizure duration is the time from reaching the Racine score of grade 1 to the end of the seizures. Values represent mean ± SE; *n* = 6 in each group. ^∗^*p* < 0.05 vs. epilepsy group.

**Figure 5:** Representative images showing pathological changes in cortex tissue of the rat brain in different groups (×400, arrows indicate the damaged cells). (a) Control group. (b) Epilepsy group. (c) Sodium valproate group. (d) GAA group. (e) The quantitative analysis of neurons' damaged rate based on the damaged nerve cells to total nerve cells in six observed fields per rat from each group. Values represent mean ± SE; *n* = 6 in each group.

**Figure 6:** Representative images showing pathological changes in hippocampal tissue of the rat brain in different groups (×400, arrows indicate the damaged cells). (a) Control. (b) Epilepsy. (c) Sodium valproate. (d) GAA. (e) The quantitative analysis of neurons' damaged rate based on the damaged nerve cells to the total nerve cells in six observed fields per rat from each group. Values represent mean ± SE; *n* = 6 in each group.

**Figure 7:** Representative immunohistochemistry micrographs of the TUNEL assay on apoptosis in cortical tissue of the rat brain (magnification ×400). Arrow indicates the apoptosis neuron. (a) Control. (b) Epilepsy. (c) Sodium valproate. (d) GAA. (e) The quantitative analysis from these images for apoptosis rate. Values represent mean ± SE; *n* = 6 in each group. In the *x*-axis of (e), A indicates control, B indicates epilepsy, C indicates sodium valproate, and D indicates GAA. ^∗∗^*p* < 0.01 vs. control group, ^##^*p* < 0.01 vs. epilepsy group.

**Figure 8:** Representative immunohistochemistry micrographs of cortical tissues from different groups (arrow indicates the changes, original magnification ×400). (a) Control. (b) Epilepsy. (c) Sodium valproate. (d) GAA. Representative analysis of expression of Bcl-2 protein in hippocampus tissue of the Western blot assay (e). Values represent mean ± SE; *n* = 6 in each group. ^∗^*p* < 0.05 vs. control group, ^#^*p* < 0.05 vs. epilepsy group.

**Figure 9:** Representative immunohistochemistry micrographs of Bax protein in cortical tissues from different groups (arrow indicates the changes, original magnification ×400). (a) Control. (b) Epilepsy. (c) Sodium valproate. (d) GAA. (e) Representative analysis of expression of Bax protein in hippocampus tissue of the Western blot assay; values represent mean ± SE; *n* = 6 in each group. ^∗^*p* < 0.05 vs. control group, ^#^*p* < 0.05 vs. epilepsy group.

**Figure 10:** Representative immunohistochemistry micrographs of cortical tissues from different groups (arrow indicates the changes, original magnification ×400). (a) Control. (b) Epilepsy. (c) Sodium valproate. (d) GAA. (e) Representative analysis of expression of caspase-3 protein in hippocampus tissue of the Western blot assay; values represent mean ± SE; *n* = 6 in each group. ^∗^*p* < 0.05 vs. control group, ^#^*p* < 0.05 vs. epilepsy group.

**Figure 11:** Effect of GAA treatment on the expression of CaSR (a), p-ERK (b), p-JNK (c), and p-P38 (d) in hippocampus tissue of the Western blot assay. Values in bottom figures represent mean ± SE; *n* = 6 in each group. In top figures and the *x*-axis of bottom figures, A indicates control, B indicates epilepsy, C indicates sodium valproate, and D indicates GAA. ^∗∗^*p* < 0.01 vs. control group, ^∗^*p* < 0.05 vs. control group, ^##^*p* < 0.01 vs. epilepsy group, and ^#^*p* < 0.05 vs. epilepsy group.

## Data Availability

Data are available upon request to the corresponding author.
